# Prediction of Geological Parameters during Tunneling by Time Series Analysis on In Situ Data

**DOI:** 10.1155/2021/3904273

**Published:** 2021-10-11

**Authors:** Shanglin Liu, Kaihong Yang, Jie Cai, Siyang Zhou, Qian Zhang

**Affiliations:** ^1^Key Laboratory of Modern Engineering Mechanics, Tianjin University, Tianjin 300072, China; ^2^Design and Research Institute of Tunneling Machine, China Railway Construction Heavy Industry, Changsha 410100, China

## Abstract

A tunnel boring machine (TBM) is a type of heavy load equipment that is widely used in underground tunnel construction. The geological conditions in the tunneling process are decisive factors that directly affect the control of construction equipment. Because TBM tunneling always takes place underground, the acquisition of geological information has become a key issue in this field. This study focused on the internal relationships between the sequential nature of tunnel in situ data and the continuous interaction between equipment and geology and introduced the long short-term memory (LSTM) time series neural network method for processing in situ data. A method for predicting the geological parameters in advance based on TBM real-time state monitoring data is proposed. The proposed method was applied to a tunnel project in China, and the *R*^2^ of the prediction results for five geological parameters are all higher than 0.98. The performance of the LSTM was compared with that of an artificial neural network (ANN). The prediction accuracy of the LSTM was significantly higher compared with that of the ANN, and the generalization and robustness of LSTM are also better than those of ANN, which indicates that the proposed LSTM method could extract the sequence properties of the in situ data. The rule of equipment-geology interaction was reflected by increasing the memory structure of the model through the introduction of the “gate” concept, and the accurate prediction of geological parameters during tunneling was realized. Additionally, the influence of time window and distance of prediction on the model is discussed. The proposed method provides a new approach toward obtaining geological information during TBM construction and also provides a certain reference for the effective analysis of the in situ data with sequence properties.

## 1. Introduction

With the rapid development of sensing technology, variety of large engineering equipment are using a large number of sensors to monitor hundreds of equipment operating parameters in real time during service. The effective analysis and modeling of in situ data are helpful in realizing the intelligent perception and prediction of the service environment and the equipment's working state.

The tunnel boring machine (TBM) is a heavy-duty equipment with high construction efficiency and safety and is widely used in modern tunnel construction. Additionally, TBM tunneling is a process relying on the rotation of the cutter head and continuously interacts with the geology ahead. Therefore, the geological conditions are the most critical influencing factor throughout the equipment's entire construction process and are the most important reference for TBM control and decision-making, which are directly related to the construction efficiency and safety. However, the TBM is underground during tunneling, and excavating interface is not visible. Therefore, the acquisition of geological information has become a key issue that is difficult to solve.

A commonly used method is drilling geological detection, which means that some exploration holes are arranged in the planned route, and the geological information is obtained by geotechnical tests. In recent years, various other geological detection methods for TBM construction have been proposed, for example, the methods using seismic waves [1–3]; the bore-tunneling electrical ahead monitoring (BEAM) technology based on electrical measurement [4]; the ground-penetrating radar (GPR) [5] method; and the advanced prediction model of the tunnel geological radar based on the cluster computing [6]. The above methods require either to be carried out before construction [7–9], or to interrupt the construction, or to install a large number of special detection devices for TBM.

Nowadays, TBM tunneling equipment generally carries a large number of sensors, and during the tunneling process, hundreds of equipment airborne parameters, such as the advance rate (AR), revolution per minute (RPM), cutter-head torque (*T*), and total thrust (*F*), can be monitored in real time. The monitoring data of these parameters can fully reflect the operating status of the equipment in real time. Since TBM tunneling is a process of continuous interaction between the equipment and the surrounding geology, the changes in the geology during tunneling are also reflected in the changes of the airborne monitoring parameters [10–13]. Therefore, the relationship between monitoring parameters and geology can be described by data analysis. However, the coupling relationship of many parameters in the monitoring data and the high-dimensional characteristics of the data make it difficult to analyze these data using simple statistical analysis methods [14, 15]. These factors make the analysis of such data challenging.

In recent years, rapidly developing information analysis methods, such as machine learning, have provided powerful tools for analyzing engineering monitoring data. Various studies have carried out basic analysis of relationship between the airborne monitoring parameters and the geological parameters based on machine learning methods. Many of these studies have established predictive models for control parameters by analyzing this relationship. For example, Mahdevari et al. [16] developed a regression model to predict penetration rate of TBM in hard rock conditions based on support vector regression (SVR). Other studies have shown that the tunneling monitoring data have the characteristics of sequence [17], and researchers used the long short-term memory (LSTM) neuron network related to time series to analyze the TBM tunneling monitoring data. For example, Gao et al. [17] proposed a TBM penetration rate (PR) prediction model based on LSTM. Li et al. [18], in order to predict the performance of the TBM, developed a long short-term memory model to predict the total thrust and the cutter-head torque of TBM in a real-time manner. In addition, some scholars have tried to classify and identify geology by analyzing the relationship between airborne parameters and geological parameters. For example, Wang et al. [19] used the extreme gradient boosting (XGBoost) algorithm to establish a model for predicting the level of the rock around the TBM. Galende-Hernández et al. [20] considered the rotation speed and penetration rate to perform the unsupervised clustering of geology and predict the rock mass rating (RMR). Culí et al. [21] considered the cutting wheel torque, penetration rate, and other parameters to assess the surrounding hydrological characteristics.

The above-mentioned studies indicate that airborne data contain important information about geology and demonstrate the feasibility of using machine learning method to analyze and extract this kind of information. However, the existing works related to geological information mainly aimed to use historical construction data to identify and classify the geology. The underground environment during TBM construction process is sophisticated, and the geological characteristics in front of the tunneling face continuously change during the entire tunneling process [22]. A kind of research demand for tunneling construction is to predict the specific future geological parameters in front of the excavation interface during the tunneling process. With the increasing distance of TBM continuous construction, the geological changes during construction are more obvious, and this demand is increasingly urgent. Therefore, how to analyze and model the monitoring data on the basis of matching the essential characteristics of the problem to realize the real-time prediction of the geology during tunneling is a key problem that needs to be solved.

Aiming at the above research demand of the engineering problems, this paper analyzed and seized the characteristics of continuity in the interaction between equipment and geology and proposed a method for the prediction of geological parameters based on the time series analysis of the monitoring data. In this paper, we make the following contributions:

1. Considering the sequence characteristics of TBM in situ data and geology, the LSTM neural network with time series analysis ability was selected, and the various parameters recorded during the TBM construction were analyzed to predict the geological parameters of the unexcavated part of the tunnel.
2. The proposed method was applied to the in situ dataset of a subway project in China, and the learning and prediction of five geological parameters, including the bulk density, cohesion, static earth pressure coefficient, internal friction angle, and elastic modulus, were carried out.
3. The prediction results obtained by the LSTM method were compared with the results obtained by the artificial neural network (ANN) method under identical conditions, and the rationality of using LSTM in geological prediction problems is explained from the viewpoints of accuracy, generalization, and robustness.
4. The influence of the time window and the distance of the advance prediction of the geological parameters on the proposed method was investigated, and the rationality of the results was analyzed based on theoretical knowledge.

The remainder of the paper is organized as follows: Section 2 explains the reasons for selecting the LSTM method for geological prediction based on theoretical analysis and the problem characteristics. The principle of this method and the specific process of its application are briefly introduced.  Section 3 presents an overview of the in situ dataset used in this study, the prediction results of the LSTM method, the comparative analysis of the LSTM method and the ANN method, and the analysis of the influence of the time window and distance of the advance prediction on the prediction results.  Section 4 summarizes the main findings and significance of this study.

## 2. Methods

### 2.1. Analysis of Geological Prediction of TBM Tunneling

Geological prediction during TBM construction is a process of predicting the unknown geology ahead of the construction by using the TBM monitoring parameters obtained from the excavated sections to construct appropriate models. The TBM construction is an orderly process [17], and the collected in situ data have a sequential nature. Otherwise, owing to the characteristics of the continuity of the TBM construction, the geology passed by the TBM is continuous; that is, the current geology is affected by the previous and, in turn, affects the subsequent geology. Therefore, to accurately predict the geological parameters, it is necessary to extract the time series information from the in situ data.

In the actual construction process, the prediction of geological parameters is also sequential; that is, as the TBM advances, the forward geology must be continuously predicted. Moreover, at the current moment, only the information of the excavated section can be used to predict the subsequent geology. Hence, practical applications cannot use data for the entire construction section to train a model. According to this characteristic, Seker and Ocak [23] proposed that when using machine learning methods to solve TBM engineering problems, attention should be paid to the division of data into training and test data and to model evaluation methods.

However, regardless of using machine learning or an empirical formula method for solving TBM problems, the relevant methods strongly rely on a complete data set that fully reflects the information of specific working conditions. Existing studies on using in situ data to solve the TBM problem often randomly shuffle the data set before training and evaluating a model [24–27]. Hence, it is difficult to obtain the preferable generalization in some projects with long span or complex environment using a learner trained on data obtained for a single construction section. Unlike the overfitting phenomenon caused by overlearning that results from noise or overparameter setting in general, the reason for the above-mentioned problem is that the training set and test set do not have the same distribution, owing to the bias of TBM data acquisition during the construction process. In other words, the construction planning and the geology passing through by TBM are a continuous and dynamic change process. Therefore, the acquisition of the airborne monitoring parameters of the TBM in the construction process does not satisfy the required randomness. The airborne monitoring parameters and the geological parameters for some sections may not represent all of the information of a project. Thus, it is possible that, even in the same project, the parameter relationship extracted from the collected data using the machine learning method may not be applicable to the subsequent construction, which greatly reduces the practical application ability of machine learning in TBM construction.

Therefore, it is necessary to introduce a method capable of time series analysis for geological prediction. However, owing to the nonstationarity and long sequence of the airborne monitoring parameters of the TBM, it is difficult to satisfy the prerequisites of conventional time series analysis [28]. Effectively mining the sequence rule is still a challenging problem in TBM data analysis.

### 2.2. LSTM Neural Network

With the increasing demand for sequence analysis and the continuous development of machine learning, new methods are constantly being proposed for time sequence analysis. Among them, the LSTM, which was developed based on the ANN and recurrent neural network (RNN), is a particular type of deep learning neural network [29]. Van Houdt et al. [30] presented a comprehensive review that covers the formulation and training of the LSTM, the relevant applications reported in the literature, and code resources implementing this method for a toy example. This method has been widely used in many fields; for example, Rehman et al. [31] proposed a novel approach, which was based on a combination of convolutional neural network (CNN) and attention-based gated recurrent unit (GRU, similar to LSTM) model, to detect single intrusion attacks as well as mixed intrusion attacks on a controller area network (CAN) bus. Ma et al. [32] proposed a LSTM-based model to tackle the missing value problem in building energy data. Hsueh and Yang [33] used a LSTM network to analyze sequential sensor data and predict the car speed of the next time interval on a freeway. Wang et al. [34] proposed a LSTM-based model that is capable of predicting the tunnel face pressure in a given operation and changing geology.

The LSTM method introduces the “gate” concept based on the RNN, which effectively solves the long-term dependence problem caused by gradient explosion or disappearance in the traditional RNN method. By using the LSTM method to process TBM data with long sequence characteristics, the long-term sequence information existing in the TBM data can be accurately learned, and existing construction data can be used to predict the geology ahead of the construction when the TBM has not completed the construction. Therefore, this study selected the LSTM method as a tool for realizing the prediction of the geological parameters in front of the tunneling construction. The most important difference between the LSTM and a classic neural network is that the LSTM neuron adds the input gate, forget gate, and output gate, which add a memory structure to the model. The basic structure of the LSTM neuron is shown in Figure 1.

In Figure 1, *C*_*t*_ represents the current cell state of the LSTM neuron, and ${\tilde{C}}_{t}$ represents the candidate information used to update the current cell state. The three gates *i*_*t*_, *f*_*t*_, and *o*_*t*_ represent input gate, forget gate, and output gate of the current neuron, respectively, and they are responsible for regulating the flow of information in and out of the current neuron. The input gate *i*_*t*_ is responsible for adding information to the neuron, and the current candidate information in ${\tilde{C}}_{t}$ can be selectively “memorized” by the LSTM neuron through the input gate. The purpose of the forget gate *f*_*t*_ is mainly to selectively forget the cell state of the previous neuron and delete information that the model considers to be unimportant. The output gate *o*_*t*_ is responsible for taking the useful information in the current cell state *C*_*t*_ as the output of the current neuron. The current candidate information ${\tilde{C}}_{t}$ and the three gates *i*_*t*_, *f*_*t*_, and *o*_*t*_ of the LSTM neuron can be calculated using equation (1) [34, 35] with similar forms:

(1) $$\begin{array}{c} {\tilde{C}}_{t}=\tanh\left(W_{C}\cdot \left[h_{t-1},x_{t}\right]+b_{C}\right),\\ i_{t}=\sigma \left(W_{i}\cdot \left[h_{t-1},x_{t}\right]+b_{i}\right),\\ f_{t}=\sigma \left(W_{f}\cdot \left[h_{t-1},x_{t}\right]+b_{f}\right),\\ o_{t}=\sigma \left(W_{o}\cdot \left[h_{t-1},x_{t}\right]+b_{o}\right). \end{array}$$

In the four formulas of equation (1), *σ* (·) and tanh(·) are the sigmoid and hyperbolic tangent functions, respectively, and · denotes the element-wise multiplication; *x*_*t*_ denotes the input data of the current neuron, and *h*_*t*−1_ denotes the hidden state of the previous neuron; *W*_*C*_, *W*_*i*_, *W*_*f*_, and *W*_*o*_ denote the weight matrix corresponding to the current candidate information ${\tilde{C}}_{t}$, input gate *i*_*t*_, forget gate *f*_*t*_ and output gate *o*_*t*_, respectively; *b*_*C*_, *b*_*i*_, *b*_*f*_, and *b*_*o*_ denote the corresponding bias terms, and these parameters need to be obtained by training the model. From equation (1), it can be seen that the current candidate information ${\tilde{C}}_{t}$ and the three gates *i*_*t*_, *f*_*t*_, and *o*_*t*_ are all determined by the output *h*_*t*−1_ of the previous neuron and the current input *x*_*t*_.

The current cell state *C*_*t*_ is the result of the cell state *C*_(*t*−1)_ of the previous LSTM neuron passing through the current forget gate *f*_*t*_ plus the current candidate information ${\tilde{C}}_{t}$ passing through the current input gate *i*_*t*_, which is expressed [35] as

(2) $$\begin{array}{c} C_{t}=f_{t}\cdot C_{t-1}+i_{t}\cdot {\tilde{C}}_{t}. \end{array}$$

At this time, the output *h*_*t*_ of the LSTM neurons, which is the result of the current cell state *C*_*t*_ processed by the activation function and then passed through the current output gate *o*_*t*_, can be expressed as [35]:

(3) $$\begin{array}{c} h_{t}=o_{t}\cdot \tanh\left(C_{t}\right). \end{array}$$

Figure 2 is a schematic diagram of the structure of the LSTM neural network. Figure 2 shows that a neuron in the LSTM neural network will transmit two states: cell state (*C*_(*t*)_) and hidden state (*h*_(*t*)_) to the next neuron. The cell state is the current state of the LSTM neuron, and the hidden state is the output of the current LSTM neuron described in Figure 1. Generally, the cell state changes slowly in the process of LSTM neural network information transmission, and the hidden state tends to be very different in different neuron nodes. The output *y*_*t*_ of the entire LSTM neural network in Figure 2 is obtained by some mapping of the output *h*_*t*_ of the last LSTM neuron.

### 2.3. Prediction of Geological Parameters Based on LSTM

The proposed method based on LSTM uses the airborne monitoring data of the TBM's performance and the geological label information accumulated in the current and previous rings as the input to predict the geological parameters of the following ring. The airborne monitoring parameters used to evaluate the construction performance of the TBM under different geological conditions include the total thrust (*F*), cutter-head torque (*T*), cutter-head revolution per minute (RPM), and the advance rate of the machine (AR) [36]. The total thrust pushes the machine forward, while the cutter-head torque sustains the constant rotation of the cutter-head to excavate the geology. The cutter-head revolution per minute and the advance rate both reflect the speed status of the machine. The geological label parameters selected in this study are the five major factors that can describe geologic features, such as the strength, density, and friction characteristics. These factors are the elastic modulus (*E*), bulk density (*ρ*), cohesion (*C*), static earth pressure coefficient (*K*_0_), and internal friction angle (*φ*).

Figure 3 shows the structure of the LSTM neural network model for predicting geological parameters. The model consists of an input layer, a LSTM network layer, a fully connected layer (dense layer), and an output layer. Let us consider the prediction of geological parameters, *A*, in the *t*^th^ ring as an example (*A* denotes one of the above-mentioned five geological parameters). In this case, the input of the LSTM network layer is the data processed by the input layer, which contains the normalized data of a total of *n* rings before the *t*^th^ ring (from *x*^(*t*−*n*−1)^ to *x*^(*t*−1)^). Additionally, *x*^(*i*)^ denotes the normalized airborne parameters and geological information corresponding to the *i*^th^ ring, including the total thrust, cutter torque, cutter rotation speed, advance rate, and geological parameter *A*. Here, *n* denotes the length of the time window (timesteps), that is, the number of the previous rings as the input data. Owing to the existence of this time window, the construction data close to the current section with limited time series can be selected as the input, to avoid the adverse effects of accumulating large amounts of early data on the training of models. After receiving the data from the input layer, the LSTM network layer will extract the time series information contained in the input data and use it as the input of a fully connected layer behind. The fully connected layer is used to compress the output dimension of the LSTM network layer to a lower size. Finally, the fully connected layer is connected to the output layer, and the output layer outputs the model's prediction *y*^(*t*)^ for the geological parameter *A* of the *t*^th^ ring.

## 3. Case Study

To test the prediction performance, the proposed method was applied to a practical project. The performance of the method was compared with that of the ANN method. Additionally, the influence of the time window and the distance of the advance prediction on the prediction accuracy of the LSTM is discussed.

### 3.1. Data Overview

The dataset used in the case study was obtained in the construction interval from Shiyijing Road Station to Dazhigu West Road Station of Tianjin Metro Line 9, which is in Tianjin, China, using a TBM for tunneling. The geological conditions of the construction are those of the typical soft soil geology in northern China, and the buried depth of the investigated construction section was approximately 10–20 m. The construction equipment is an earth pressure balance (EPB) TBM machine produced by Komatsu, Japan, with a diameter of 6.34 m. The dataset used consists of geological label parameters and airborne monitoring parameters. The geological label parameters were obtained by geological exploration before the commencement of the project, and the airborne monitoring parameters were collected in real time by a variety of sensors installed on the TBM during the construction process and collated and stored by the TBM data acquisition system.  Table 1 lists the statistical properties of the key airborne monitoring parameters and the geological parameters, which are the prediction targets of the LSTM.

Owing to the different dimensions of the TBM airborne monitoring parameters and geological parameters, the magnitude difference is large. To facilitate the gradient update and accelerate the convergence of the network's training, this study carried out normalization preprocessing (Min-Max Scale) on the data in the dataset. All the airborne parameters and geological parameters were normalized for subsequent model training and testing. The calculation method is expressed as [18]

(4) $$\begin{array}{c} x_{\text{pre}}=\frac{x-x_{\min}}{x_{\max}-x_{\min}}. \end{array}$$

In equation (4), *x*_pre_ is the value of a parameter after normalization preprocessing, *x* denotes the original value of the parameter, *x*_min_ is the minimum value corresponding to the parameter in the recorded data, and *x*_max_ is the maximum value corresponding to the parameter in the recorded data.

To analyze the relationship between the selected TBM airborne monitoring parameters and geological parameters, the single independent variable linear regression relationships between four airborne monitoring parameters and five geological parameters were calculated and evaluated using coefficient of determination (*R*^2^) evaluation indicator.  Figure 4 shows the scatter plot and *R*^2^ of the linear regression between the normalized TBM performance parameters and the geological parameters. The abscissa of each subgraph represents an airborne parameter, while the ordinate represents a geological parameter. As can be seen, the scatters in all subgraphs do not exhibit a significant linear relationship.

Table 2 presents the average *R*^2^ between the four TBM airborne monitoring parameters and geological parameters. The maximum of the four average *R*^2^ is the *R*^2^ between the total thrust and the five geological parameters, which is less than 0.25, and the average *R*^2^ between the cutter-head torque and the five geological parameters was minimum, that is, only 0.004. These results confirm that there is no significant linear relationship between a single performance parameter and the geological parameters. If the airborne parameters are used to accurately predict the geological parameters, it is necessary to consider the interaction between multiple airborne parameters simultaneously, which also indicates that the use of airborne parameters for predicting the geological parameters is a complex coupling problem with multiple inputs.

### 3.2. Experimental Results

For the data of Tianjin Metro Line 9, the LSTM algorithm was used to predict the geological parameters in front of the tunneling excavation. With regard to the LSTM hyperparameters, the number of neurons in the LSTM network layer was set to 100. The size of the full connection layer was 20, and the size of the output layer was 1. Adaptive moment estimation (Adam) was used as the optimization method, and the error calculation method was the mean absolute error (MAE). Rectified linear unit (ReLU) was selected as the activation function of the full connection layer. As a crucial parameter in the LSTM, the time window was set to 5, which was used as the default value in subsequent analysis, and the reason will be explained in the analysis part later. The data set was divided into the training set and test set by order according to the ratio of 7 : 3, and these data sets were used to train and test the LSTM model established under the above-mentioned parameter settings. The test set data were not considered in the training process and were instead used to individually test the prediction effect.

Figure 5 shows the predicted curves and measured points when predicting the five geological parameters in the test set. The blue columns at the bottom of each subgraph represent the residual between the predicted value and the actual value of the geological parameters. Figure 5 also shows the histograms of the residual percentage. It can be seen from the measured points and predicted curves in Figure 5 that the points and curves of the five geology parameters are very consistent, which indicates that the proposed method can effectively predict the five geological parameters. Besides, four geological parameters, namely, the elastic modulus, bulk density, cohesion, and internal friction angle, sharply fluctuated around the ring number 800. The internal friction angle greatly fluctuated close to the ring numbers 740, 800, 850, and 930. However, the values predicted by the LSTM for these five geological parameters are still essentially consistent with the actual values in the position of large numerical fluctuations. This indicates that the constructed LSTM model can accurately predict the geological parameters when the geological parameters greatly fluctuate, and the model can accurately reflect the change trend of the geological parameters.

In addition, it can be seen from the residuals that, firstly, the residuals of the five geological parameters predicted by the LSTM method are significantly smaller than the actual values of the geological parameters, and most residuals are less than 0.5% of the measured value. Secondly, although the prediction accuracy of the LSTM method can reach a high level at a position where the geological parameters exhibit large fluctuation, it is still significantly lower than the prediction accuracy at the position of stable geological parameters. To a certain extent, this indicates that the mutation of the prediction parameters has a negative impact on the prediction effect of the LSTM model. Thirdly, except for the position where the geological parameters change to a great extent, the residuals in other places are approximately randomly distributed, and the systematic error of the model is small, which demonstrates that the LSTM can fully extract the rules contained in the time series data, and a missing factor that is closely related to the geological parameters does not exist.

To further quantitatively evaluate the performance of the LSTM method, statistical indicators including the coefficient of determination (*R*^2^), mean absolute error (MAE), and mean absolute percentage error (MAPE) were used to evaluate the performance of the LSTM model. For a given predicted value $\hat{y}=\left\{{\hat{y}}_{1},{\hat{y}}_{2},\ldots ,{\hat{y}}_{n}\right\}$, measured value *y*={*y*_1_, *y*_2_,…, *y*_*n*_}, and the average value $\bar{y}$ of $\hat{y}$, the above-mentioned evaluation indices are calculated by equations (5)–(7) [18, 34]:

(5) $$\begin{array}{c} R^{2}\left(y,\hat{y}\right)=1-\frac{\sum_{i=1}^{n}{\left(y_{i}-{\hat{y}}_{i}\right)}^{2}}{\sum_{i=1}^{n}{\left(y_{i}-\bar{y}\right)}^{2}}, \end{array}$$

(6) $$\begin{array}{c} \text{MAE}=\frac{1}{n}\sum_{i=1}^{n}\left|y_{i}-{\hat{y}}_{i}\right|, \end{array}$$

(7) $$\begin{array}{c} \text{MAPE}=\frac{1}{n}\sum_{i=1}^{n}\left|\frac{y_{i}-{\hat{y}}_{i}}{y_{i}}\right|\times 100\%. \end{array}$$

Here, *R*^2^ can reflect the proportion of the variations of the dependent variable that can be explained by the independent variable through the regression relationship; MAE is the average absolute error between the predicted and actual values, which can better reflect the actual values of the error and can be used as the loss function of the regression problem; MAPE is the average relative error between the predicted and actual values. Therefore, *R*^2^ reflects the similarity between the predicted values and the true values, and the prediction effect of the model improves as the value of *R*^2^ approaches 1. MAE and MAPE reflect the difference between the predicted values and the true values, and the prediction accuracy increases as their value becomes smaller. By recording the evaluation index information in the line chart, it can be seen that the *R*^2^ of the LSTM's prediction results for the five geological parameters are all higher than 0.98, the MAPE values are lower than 1%, and the MAE values are lower than 0.5% of the average of corresponding geological parameters.

To further analyze the applicability of the proposed method under other working conditions, this study used the LSTM method to predict five geological parameters based on the in situ dataset of another subway project in the same city, namely, Tianjin Metro Line 3. In the calculation, the dataset was divided into the training set and test set in order, according to the ratio of 7 : 3. Considering the small amount of data in this dataset, the time window was set to 2. The sizes of the LSTM network layer, full connection layer, and output layer were 100, 20, and 1, respectively. The Adam algorithm was used as the optimization method, MAE was used as the loss function, and ReLU was selected as the activation function. Moreover, the *R*^2^, MAE, and MAPE were used to evaluate the prediction effect of the model. The results reveal that the *R*^2^ of the LSTM prediction results obtained for the five geological parameters are higher than 0.86, and the average *R*^2^ reached 0.94. All MAPE values are all lower than 2%, while the MAE values are much smaller compared with the average value of the corresponding geological parameters, and lower than 2.5% of the average value of the corresponding geological parameters. The above results indicate that the LSTM method could realize the real-time and highly accurate prediction of the five geological parameters.

### 3.3. Comparative Analysis of LSTM and ANN

To reflect the superiority of the LSTM, the performance of the LSTM was compared with that of an ANN. To ensure that the ANN structure was similar to the LSTM structure, the hidden layer structure was set to (100, 20). The Adam method was used as the optimization method, MAE was used as the loss function, and ReLU was selected as the activation function. The time window of the ANN was also set to 5. The ANN model was trained by the same input data as the LSTM, and the prediction results were tested on the same test set.

Table 3 lists the indices of *R*^2^, MAE, and MAPE when the LSTM and ANN predicted the five geological parameters. It is not difficult to conclude that the prediction results obtained by the LSTM method are better in all situations compared with those of ANN. When predicting various geological parameters, the prediction accuracy of the LSTM was significantly higher compared with that of the ANN. For example, when predicting the static earth pressure coefficient, the *R*^2^ index of LSTM was 222.78% higher than that of the ANN, while the MAPE and MAE indices were only approximately 10% of those of the ANN model. The average *R*^2^ of LSTM is 0.41 higher than ANN. The MAPE and MAE of LSTM are only 15.9% and 16.2% of ANN on average, respectively. The above results indicate that, compared with ANN, the LSTM can effectively extract the temporal information in the data and is more suitable to the real-time prediction of various geological parameters.

According to the above-mentioned prediction results, Figure 6 shows the histograms of the three evaluation indices when the LSTM model and ANN model predicted five geological parameters. As can be seen from Figure 6(a), the accuracy of the LSTM model was maintained at a high level when different geological parameters were predicted. The category of the predicted geological parameters has a small effect on its prediction accuracy, and the model has good generalization. The ANN model exhibits great difference in terms of its prediction accuracy for different geological parameters and was greatly affected by the predicted geological parameters, which indicates that its generalization is poor. Figures 6(b) and 6(c) show that there are certain differences in model errors when predicting different geological parameters, but the errors of LSTM are significantly lower than those of ANN.

Furthermore, Figure 7 shows the *R*^2^ curves of five geological parameters predicted by the LSTM model and ANN model with different sizes of time windows. In this figure, the abscissa represents the size of the selected time window, and the ordinate represents the *R*^2^ of the model. As can be seen, the prediction accuracy of the LSTM model for different geological parameters was stable and less affected by the change of the time window and performed satisfactorily under different time windows. The prediction accuracy of the ANN model for different geological parameters obviously fluctuated with the change of the time window, which indicates that it is sensitive to the selection of the time window. Additionally, the time window with the highest prediction accuracy was not the same when different geological parameters were predicted by the ANN. Therefore, it is considered that the LSTM model constructed in this study has strong robustness to the setting of the time window when predicting different geological parameters, and the selection of the time window does not need to rely too much on prior knowledge. In other words, even if the time window is randomly selected, the prediction results obtained by the LSTM have high accuracy. When using the ANN model to predict different geological parameters, experiments need to be carried out separately for different geological parameters, and the optimal time window size should be selected according to the experimental results.

In summary, the above-mentioned comparison results reveal that, compared with the ANN, the LSTM has higher accuracy and stronger generalization and robustness in the prediction of geological parameters and can achieve reliable prediction of various geological parameters under different time windows.

### 3.4. Effect of Time Window and Distance of Prediction on LSTM

In order to further explore the influence of different input-output situations on the LSTM, we discussed the influence of the time window and the distance of prediction on the model accuracy in this section.

Figure 8 shows the *R*^2^ curves of the LSTM model when predicting five geological parameters under different time windows. As can be seen, when the LSTM model predicts the five geological parameters, the prediction accuracy increases with the time window at first and then slightly fluctuates at a higher level. Notably, when the time window is 5, the *R*^2^ of the five geological parameters essentially stop exhibiting an upward trend and achieve high prediction accuracy. Therefore, the default time window size was set to 5 in the proposed LSTM model. Actually, the selection of time windows is related to the size of the training set and the time series characteristics of the data.

In principle, the data that have great influence on the geological parameters of the next ring are the data of the current ring and several adjacent rings before the current ring, while the data collected earlier have little influence on the geological parameters of the next ring. Therefore, when the time window was less than 5, the data used to predict the geological parameters were all within the previous adjacent five rings, and this part of the data was strongly correlated with the geological parameters of the next ring. At this stage, the increase of the time window leads to the increase of effective information input to the model, and thus the prediction accuracy of the model increases with the time window. When the time window was greater than 5, although the increase of the time window led to the increase of the input data, the effective information input to the model did not increase. The data increased is far from the geological parameters predicted in the next ring and less related to them. So, with the continuous increase of the time window, the prediction accuracy of the model no longer changes significantly.

Figure 9 shows the histogram of *R*^2^ of the prediction results for the five geological parameters under different distances of the advance prediction when the size of the time window is 5. The abscissa of the figure represents the predicted geological parameters, and the ordinate represents the *R*^2^ of the predicted results. The columns with different colors in the graph represent different distances of the advanced prediction. In this study, the distance of the advance prediction (referred to as *Distance* in the figure) was replaced by the number of rings between the current ring and the ring to be predicted. For example, by assuming that the distance of the advance prediction is *n* rings, then, under the same input conditions, the prediction target of the LSTM model is the geological parameter of the *n*^th^ ring after the current ring.

It can be found in Figure 9 that the accuracies of the prediction results of the five geological parameters all decrease as the distance of the advance prediction increases. When the distance of the advance prediction is 1 ring (the pink columns), which is the default value used in the above-mentioned prediction, the *R*^2^ of the five geological parameter prediction results are approximately the same in the graph and are close to 1. When the distance increases to five rings (the green columns), the *R*^2^ for the bulk density prediction are already lower than zero, which indicates that the model has lost its ability to predict the bulk density at this time. When the distance of the advance prediction increases to nine rings (the purple columns), the *R*^2^ for the elastic modulus, static earth pressure, and internal friction angle have also dropped to approximately zero; that is, the model has lost its predictive ability for all five geological parameters at this time.

This demonstrates that there is an “effective distance” for predicting the geological parameters ahead of the construction using the current data. In other words, the current data can only realize the effective prediction of geological parameters within a certain range in front of the excavation. The above-mentioned results reveal that the current airborne monitoring parameters and geological parameters are closely related to the geological parameters within a short distance but have a small effect on the geological parameters farther away. This is consistent with the theory that the current construction situation is only affected by the geological conditions of the current and the limited distance ahead in the shield construction process.

## 4. Conclusion

In this study, a geological parameter prediction method based on the in situ data of TBM engineering is proposed. By considering the sequence characteristic of the TBM in situ data, the method based on the LSTM neural network was selected to analyze the time series of various parameters recorded during TBM construction, and the geological parameters in front of the tunneling excavation were subsequently predicted. The proposed method was applied to the Tianjin Metro Line 9, which is an urban subway project constructed using an EPB TBM in China. The results reveal that the real-time geological parameter prediction method based on the LSTM could realize the real-time and accurate prediction of five geological parameters, namely, the bulk density, cohesion, static earth pressure coefficient, internal friction angle, and elastic modulus.

The LSTM method was compared with an ANN model under identical conditions. The comparison results reveal that the LSTM predicted the five geological parameters with high accuracy, and the average *R*^2^ of the prediction results for the five geological parameters was higher than 0.98, which is significantly higher than that of the ANN. Moreover, the generalization and robustness of the LSTM are significantly better compared with the ANN. Additionally, the influence of the time window and the distance of the advance prediction on the accuracy of the LSTM model was also investigated. The results reveal that the *R*^2^ for the five geological parameters obtained by the proposed LSTM model increased at first, then slightly fluctuated at a high level with the increase of the time window, and decreased with the increase of the distance of the advance prediction. This indicates that the current airborne monitoring parameters and geological parameters can only reflect the geological parameters of a finite distance ahead of the construction.

The proposed method for predicting the advanced geological parameters could effectively extract the time series information from the in situ data of Tianjin Metro Line 9 and realize the accurate and real-time prediction of the geology in front of the tunneling excavation. Finally, the proposed method provides a reference for the processing of in situ data with sequence properties, such as TBM parameters.

## Figures and Tables

**Figure 1:** Schematic diagram of the LSTM neuron structure. The LSTM neuron contains states, gates, inputs, and outputs.

**Figure 2:** The structure of the LSTM neural network.

**Figure 3:** Structure of the LSTM neural network model for geological prediction.

**Figure 4:** Relationship between airborne monitoring parameters and geological parameters.

**Figure 5:** LSTM prediction results for different geological parameters. (a) Elastic modulus. (b) Bulk density. (c) Cohesion. (d) Static earth pressure coefficient. (e) Internal friction angle.

**Figure 6:** Results for five geological parameters predicted by ANN and LSTM under different indices. (a) *R*^2^ of predictions. (b) MAPE of predictions. (c) MAE of predictions.

**Figure 7:** *R* ^2^ of ANN and LSTM for prediction of different geological parameters in different time windows. (a) The prediction of elastic modulus. (b) The prediction of bulk density. (c) The prediction of cohesion. (d) The prediction of static earth pressure coefficient. (e) The prediction of internal friction angle.

**Figure 8:** *R* ^2^ of LSTM model predicting different geological parameters under different time windows.

**Figure 9:** *R* ^2^ of LSTM model predicting different geological parameters with different distances of advanced prediction.

**Table 1:** Basic statistical properties of in situ data used in Tianjin metro line 9.

Parameter	Symbol	Unit	Max	Min	Avg	Std
Advance rate	AR	mm/min	55.68	16.84	35.23	10.04
Thrust force	*F*	kN	24701.68	10436.07	15840.43	2905.33
Cutter-head torque	*T*	kNm	1706.28	803.08	1264.49	148.71
Revolution per minute	RPM	rev/min	1.10	0.40	0.94	0.14
Elastic modulus	*E*	MPa	7.89	4.70	6.57	0.52
Bulk density	*ρ*	g/cm^3^	2.23	1.60	2.10	0.06
Cohesion	*C*	kPa	32.93	19.84	28.03	2.10
Static earth pressure coefficient	*K*_0_	—	0.45	0.32	0.40	0.03
Internal friction angle	*φ*	°	22.98	14.05	19.53	1.76

**Table 2:** Average *R*^2^ between various performance parameters and geological parameters.

	AR (mm/min)	*F* (kN)	*T* (kNm)	RPM (*r*/min)
Ave *R*^2^	0.140	0.236	0.004	0.105

**Table 3:** Prediction results of different geological parameters by LSTM and ANN under different evaluation indices. The best result is highlighted in bold.

Geologic parameter	Evaluation index	ANN	LSTM
Elastic modulus	*R* ^2^	0.5688	**0.9883**
	MAPE	0.0317	**0.0050**
	MAE	0.1862	**0.0299**

Bulk density	*R* ^2^	0.5945	**0.9859**
	MAPE	0.0131	**0.0018**
	MAE	0.0246	**0.0034**

Cohesion	*R* ^2^	0.7357	**0.9914**
	MAPE	0.0256	**0.0053**
	MAE	0.6670	**0.1433**

Static earth pressure coefficient	*R* ^2^	0.3051	**0.9848**
	MAPE	0.0273	**0.0035**
	MAE	0.0111	**0.0014**

Internal friction angle	*R* ^2^	0.6780	**0.9906**
	MAPE	0.0399	**0.0066**
	MAE	0.6722	**0.1141**

## Data Availability

The data used in this paper are from the relevant engineering enterprises, which have not been released for commercial reasons.
